# Health Evaluation and Fault Diagnosis of Medical Imaging Equipment Based on Neural Network Algorithm

**DOI:** 10.1155/2021/6092461

**Published:** 2021-09-04

**Authors:** Zhenwei Zhao, Weining Jiang, Weidong Gao

**Affiliations:** ^1^Information Center of the First Hospital of Jilin University, Changchun 130021, Jilin, China; ^2^School of Information and Communication Engineering, Beijing University of Posts and Telecommunications, Beijing 100876, China

## Abstract

In recent years, high-precision medical equipment, especially large-scale medical imaging equipment, is usually composed of circuit, water, light, and other structures. Its structure is cumbersome and complex, so it is difficult to detect and diagnose the health status of medical imaging equipment. Based on the vibration signal of mechanical equipment, a PLSR-DNN hybrid network model for health prediction of medical equipment is proposed by using partial least squares regression (PLSR) algorithm and deep neural networks (DNNs). At the same time, in the diagnosis of medical imaging equipment fault, the paper proposes to use rough set to screen the fault factors and then use BP neural network to classify and identify the fault and analyzes the practical application effect of the two technologies. The results show that the PLSR-DNN hybrid network model for health prediction of medical imaging equipment is basically consistent with the actual health value of medical equipment; medical imaging equipment fault diagnosis technology is based on rough set and BP neural network. In the test set, the sensitivity, specificity, and accuracy of medical imaging equipment fault identification are 75.0%, 83.3%, and 85.0%. The above results show that the proposed health prediction method and fault diagnosis method of medical imaging equipment have good performance in health prediction and fault diagnosis of medical equipment.

## 1. Introduction

With the development of science, modern mechanical equipment has entered a new stage, and more and more mechanical equipment has entered people's daily life [1]. With the development of new technology of medical equipment, a large number of high-precision and highly mechanized medical imaging equipment have entered various hospitals [2]. With the influx of a wide range of medical imaging equipment into the hospital, how to carry out the scientific and effective management of these medical imaging equipment is imminent [3]. The basic link of medical imaging equipment management is the evaluation of medical imaging equipment health and the diagnosis of medical imaging equipment fault [4]. At this stage, the skill level of medical technicians in professional maintenance and testing of medical imaging equipment still needs to be improved, and it is difficult to achieve the synchronous improvement of medical imaging equipment technology [5, 6]. In other words, the failure of medical imaging equipment inventory has become the difficulty of medical imaging equipment management. In view of this, this paper proposes to mine the influencing factors of medical imaging equipment fault through rough set, describe the medical imaging equipment universe data set with information table, and find out the condition attribute and decision attribute in different medical equipment. In the case of maintaining the primary category of rough set, we reduce the redundant data in rough set, that is, we retain really useful data by reducing dimension. Then, the BP neural network is used to identify and classify the fault factors to complete the medical imaging equipment fault diagnosis. In the aspect of health evaluation of medical equipment, the parameters associated with the health of medical imaging equipment are extracted as the input features of the health prediction model. Partial least squares regression algorithm (PLSR) neural network and deep neural network (DNN) PLSR-DNN hybrid neural network model are constructed.

Meng et al. proposed a multifeature fusion fault diagnosis method based on the combination of quadratic filter and QPSO-KELM algorithm. It has achieved excellent diagnosis results in gearbox fault diagnosis. Guo et al. used the belief network of parameter optimization to diagnose the bearing fault. The diagnosis results show that the method can correctly identify the bearing faults under different conditions, greatly improve the intelligence of fault classification, and reduce the time of parameter selection of deep learning model [7]. The two-dimensional visualization of the original acoustic emission signal has been used by scholars such as Islam and Kim to provide bearing health information [8]. Han et al. believe that in-depth learning has become a new research direction in the field of intelligent monitoring and fault diagnosis of industrial equipment [9]. In order to improve the diagnosis accuracy of the mechanical equipment fault diagnosis model, Tang and other scholars proposed a fault diagnosis model of mechanical equipment with feature selection feedback network [10]. Wang and other scholars proposed a fault diagnosis model of mechanical equipment based on noise assisted signal enhancement and stochastic resonance and optimized the parameters by particle swarm optimization. Ma et al. put forward that rolling bearing is the key component of mechanical equipment, and it plays an important role in fault detection of mechanical equipment.

Reid et al. believe that it is necessary to pay attention to the fault diagnosis of sterilization pod, especially in Africa [11]. Bebronne and other scholars used artificial neural network (ANN) and partial least squares regression (PLSR) to estimate the area under the infection progress curve in the study of winter wheat fungal infection [12]. Perin et al. used partial least squares regression (PLSR) and spectrophotometry combined with color image and spectrophotometry to evaluate the antioxidant activity of *Picea asperata* [13]. Kristoffersen and other scholars have established a partial least squares regression (PLSR) model to predict DH% by molecular weight distribution to predict the degree of hydrolysis of milk protein hydrolysate [14]. Shen et al. believe that light, near infrared and mid infrared reflectance spectra combined with partial least squares regression method is an effective method to determine soil properties [15]. Dong and other scholars improved the residual of multiple linear regression model by partial least squares regression and support vector regression [16]. Meunier et al. believe that partial least squares regression (PLSR) can predict the contribution of electrochemical drift to subsequent full voltammetric scanning [17]. Sun et al. and other researchers proposed a power system asset fault prediction scheme combining unsupervised and supervised learning, and the experimental results show that it has good performance [18].

To sum up, in recent years, there are a lot of research studies on artificial neural network, partial least squares regression, mechanical equipment fault, and so on, but the research on health evaluation and fault diagnosis prediction of medical imaging equipment through neural network is relatively lacking. Therefore, a medical imaging equipment health evaluation technology based on PLSR-DNN hybrid neural network and a medical imaging equipment fault diagnosis technology based on rough set and BP neural network are proposed to assist people in the evaluation and diagnosis of medical imaging equipment health and fault.

## 2. Research on the Health Evaluation and Fault Diagnosis Method of Medical Imaging Equipment Based on Neural Network Algorithm

### 2.1. Health Evaluation Technology of Medical Imaging Equipment Based on Neural Network Algorithm

Firstly, the parameters related to the health status of medical imaging equipment are extracted by calculating the characteristic parameters of the vibration signal characterization signal, which are used as the input characteristics of the health degree prediction model [19]. When the medical machinery is in the same healthy state, its vibration signal belongs to stable signal [20].

(1) $$\begin{array}{c} \frac{1}{j-i}\int_{t_{i}}^{t_{j}}V_{k}\left(t\right)\text{d}t=M\approx C_{1}, \end{array}$$

(2) $$\begin{array}{c} \frac{1}{j-i}\int_{t_{i}}^{t_{j}}{\left(V_{k}\left(t\right)-M\right)}^{2}\text{d}t=S\approx C_{2}. \end{array}$$

Expressions (1) and (2) indicate the *i* vibration signal sampling point in the working period *T*_*k*_ of medical machinery with health degree *k*, where *i*=1,2,… of *t*_*i*_ and health degree is *k*=1,2,…. *V*_*k*_(*t*) represents the vibration signal, which refers to the amplitude of the vibration signal corresponding to the medical imaging equipment with *k* health degree collected at a time. The mean value and standard deviation of vibration signal in *t*_*i*_ ~ *t*_*j*_ period are *M* and *S*, respectively. *C*_1_, *C*_2_ are constants, and both of them are only affected by health degree *k*. With the use of medical equipment, its health gradually degenerates, and the overall performance of vibration signal is nonstationary signal [21]. The characteristic frequencies of different parts of mechanical equipment are different, and the amplitude frequency form of vibration signal *a*(*f*) can be obtained by the time-frequency conversion tool.

(3) $$\begin{array}{c} \text{s.t. }\phi_{n}=\left[f_{i},f_{j}\right]\left(f_{i}<f_{j}\right), \end{array}$$

where *f*_*i*_ represents *i* frequency points and *ϕ*_*n*_ represents *n* continuous frequency interval corresponding to the first characteristic frequency. ∀*f*_*n*_ ∈ *ϕ*_*n*_, *a*(*f*_*n*_) − *η*^+^ > 0, *η*^+^=*μ*+*γσ*, in which *η*^+^=*μ*+*γσ* is mainly responsible for the detection of signal outliers, *η*^+^ refers to the average level, which is used to determine the size of continuous frequency interval, *μ* is the mean value of the signal, *σ* refers to the standard deviation of the signal, and *γ* ∈ [3, +*∞*) is the factor responsible for determining the positive average [22, 23].

(4) $$\begin{array}{c} A^{*}=\left\{a\left(f_{1}^{*}\right),a\left(f_{2}^{*}\right),\ldots ,a\left(f_{n}^{*}\right)\right\}, \end{array}$$

where *A*^*∗*^ represents the amplitude of the characteristic frequency corresponding to the extracted vibration signal and *A*^*∗*^ is the frequency domain. *f*_*n*_^*∗*^=argmax_*f*_*n*_∈*ϕ*_*n*__{*a*(*f*_*n*_)}, where *f*_*n*_^*∗*^ represents the *n* characteristic frequency. So, the equivalent calculation of *M*, *S*, *A*^*∗*^ does not depend on the physical structure and failure mechanism of medical equipment, so it can analyze different types of vibration signals [24].

The partial least squares regression algorithm is introduced to select features from the linear level (PLSR), and the nonlinear level regression mapping between the selected features and the health degree of medical imaging equipment is established through the deep neural network (DNN), so as to construct the PLSR-DNN hybrid neural network health degree prediction model [25].

As shown in Figure 1, PLSR-DNN model is composed of PLSR layer and DNN layer. The former uses PLSR to carry out linear regression mapping on input features, while the latter uses DNN to carry out nonlinear regression mapping on output of the first layer, where *M*, *S*, *A*^*∗*^ belong to a medical imaging equipment through vibration signal acquisition *n*. The average value of each characteristic is 0, and the variance is 1.

(5) $$\begin{array}{c} X_{0}=\left[x_{1}^{T},x_{2}^{T},\ldots ,x_{n}^{T}\right], \end{array}$$

(6) $$\begin{array}{c} Y_{0}=\left[y_{1}^{T},y_{2}^{T},\ldots ,y_{m}^{T}\right], \end{array}$$

where *X*_0_ represents the input data matrix with *n* vibration signal features and *Y*_0_ represents the target data matrix with *m* health labels. The input sample vector with *m* data is represented as *x*^*T*^. The target sample vector with *m* data is represented as *y*^*T*^. According to the data matrix, the space projection is started:

(7) $$\begin{array}{c} t_{1}=x_{1}w_{11}+x_{2}w_{12}+\cdots +x_{n}w_{1n}=X_{0}w_{1}, \end{array}$$

(8) $$\begin{array}{c} u_{1}=y_{1}v_{11}+y_{2}v_{12}+\cdots +y_{m}v_{1m}=Y_{0}v_{1}, \end{array}$$

where *t*_1_ represents the linear combination of input sample vectors; *u*_1_ is the linear combination of the target sample vectors; the *n* element of the unit vector *w*_1_ is *w*_1*n*_; the *m* element of the unit vector *v*_1_ is *v*_1*m*_; the eigenvector of *X*_0_^*T*^*Y*_0_*Y*_0_^*T*^*X*_0_ is *w*_1_; and the eigenvector of *Y*_0_^*T*^*X*_0_*X*_0_^*T*^*Y*_0_ is *v*_1_. When the spatial correlation of *t*_1_ and *u*_1_ after projection reaches the maximum, there is *t*_1_ ≈ *u*_1_. The regression models of *X*_0_ and *Y*_0_ to *t*_1_ were established:

(9) $$\begin{array}{c} \left\{\begin{array}{c} X_{0}=t_{1}\alpha_{1}+E_{1},\\ Y_{0}=t_{1}\beta_{1}+F_{1}, \end{array}\right) \end{array}$$

where *α*_1_, *β*_1_ represent parameter vectors and *E*_1_, *F*_1_ represent residual matrix. When there is a rank of matrix *X*_0_ is *r*, there are as follows:

(10) $$\begin{array}{c} X_{0}=t_{1}\alpha_{1}+t_{2}\alpha_{2}+\cdots t_{r}\alpha_{r}+E_{r}, \end{array}$$

(11) $$\begin{array}{c} Y_{0}=t_{1}\beta_{1}+t_{2}\beta_{2}+\cdots t_{r}\beta_{r}+F_{r}, \end{array}$$

where *α*_*i*_(*i*=1,2,…, *r*), *β*_*i*_(*i*=1,2,…, *r*) are parameter vectors (*α*_*i*_=*X*_0_^*T*^*t*_*i*_/‖*t*_*i*_‖^2^, *β*_*i*_=*Y*_0_^*T*^*t*_*i*_/‖*t*_*i*_‖^2^, and *t*_*i*_=*X*_0_*w*_*i*_(*i*=1,2,…, *r*)) and *E*_*r*_, *F*_*r*_ represent the minimum residual matrix.

(12) $$\begin{array}{c} Y_{0}=X_{0}w_{1}\beta_{1}+X_{0}w_{{}_{2}}\beta_{2}+\cdots X_{0}w_{r}\beta_{r}+F_{r}. \end{array}$$

Equation (12) is the PLSR equation, which is responsible for processing input variables in the linear mapping layer when predicting the health of medical equipment and can effectively reduce the difficulty of network optimization.

Figure 2 shows a deep neural network with two hidden layers. The neurons in the adjacent layers are fully connected with each other. *x*_*i*_(*i*=1,2,…, *n*) is the input characteristic of the vibration signal of the medical imaging equipment after PLSR processing; $\hat{y}$ indicates the health prediction output of medical equipment; Relu is selected as the activation function between the hidden layers; and linear output is selected between the hidden layer and the output layer.

(13) $$\begin{array}{c} J\left(W,b\right)=\frac{1}{m}\sum_{i=1}^{m}L\left({\hat{y}}^{i},y^{i}\right)=\frac{1}{m}\sum_{i=1}^{m}L{\left({\hat{y}}^{i}-y^{i}\right)}^{2}, \end{array}$$

where *W* is the weight matrix of each layer, *b* is the deviation matrix of the corresponding layer, the mean square error is selected as the loss function *J*(*W*, *b*), and *y*^*i*^ represents the actual value of the data target of group *i*. At the same time, the predicted value of group *i* is represented by ${\hat{y}}^{i}$. In order to reduce overfitting, regularization term is introduced.

(14) $$\begin{array}{c} J\left(W,b\right)=\frac{1}{m}\overset{m}{\underset{i=1}{\sum }}L\left({\hat{y}}^{i},y^{i}\right)+\frac{\lambda }{2m}{\left\|W\right\|}_{2}^{2}=\frac{1}{m}\sum_{i=1}^{m}L{\left({\hat{y}}^{i}-y^{i}\right)}^{2}+\frac{\lambda }{2m}\sum_{j=1}^{n}W_{j}^{2}\\ =\frac{1}{m}\sum_{i=1}^{m}L{\left({\hat{y}}^{i}-y^{i}\right)}^{2}+\frac{\lambda }{2m}\sum_{j=1}^{n}W^{T}W, \end{array}$$

where *λ* represents the regularization parameter and *m* represents the number of sample sets. After regularization, the deep learning network can limit the parameters to be too large or too many. After processing, the weight of each layer is set to 0.

(15) $$\begin{array}{c} H_{D}=T-T_{O}, \end{array}$$

where *H*_*D*_ indicates the current health of the medical device, *T* indicates the total operation time of medical imaging equipment before failure, and *T*_*O*_ indicates the current running time of the medical device.

### 2.2. Design of Medical Imaging Equipment Fault Diagnosis Method Based on Neural Network Algorithm

Rough set theory can mine the interaction of different fuzzy datasets from the existing data and explain the potential laws. Its core is the division of related knowledge, related sets, approximate sets, and so on [22]. As medical equipment, especially large medical equipment, is usually composed of electronic components, circuits, machinery, optical path, etc., the structure is complex and cumbersome, so it is very difficult to detect its fault, and it is difficult to describe the internal logic of medical imaging equipment with conventional methods. In the research process, the information table of rough set is used to describe the relevant data sets. We take the ventilator as an example (see Table 1).

In Table 1, the “oxygen supply concentration” is selected as the condition attribute of rough set, the “influence on respiratory therapy” factor is selected as the decision attribute of rough set, and the decision rule is found through the implied condition attribute, that is, the influence on respiratory therapy is found through the oxygen supply concentration. The reduction process of rough set is reduced to process, and only the core of rough set is retained. However, the reduction set of a rough set is not a unique set. Because the reduction process of medical imaging equipment fault factors is directly limited by software, hardware and inherent conditions of equipment, and other factors, attribute importance reduction algorithm is used to complete the reduction of rough set. In addition, in terms of generalization ability and fault tolerance ability, rough set theory has some shortcomings, so unsupervised BP neural network combined with rough set theory is used. The input dimension of neural network is simplified by rough set reduction, as shown in Figure 3.

As shown in Figure 3, after the training samples are input, the conditional attributes are quantified. The redundant items are removed according to the quantitative results, and the decision tree is constructed by using the remaining samples. The equivalence set of condition attribute and decision attribute is calculated. The importance of attributes is calculated. When the importance is 0, delete and observe whether the decision table is consistent. If it is consistent, simplify the attribute. After all the attributes have been calculated, the simplified decision table can be obtained. After rule acquisition, rule simplification, and training planning, the conditional attributes are selected, and the final classification results are output through BP neural network classification model. In addition, after the test set samples are input, the conditional attributes are quantified, the conditional attributes are selected, and the BP neural network is used to classify. Ventilator is an important life support equipment in clinical treatment, so we choose ventilator as the representative of medical imaging equipment to build the experimental model.

As shown in Table 2, it mainly collects the environmental data factors, electrical factors, and gas path factors that cause ventilator failure, among which the environmental factors refer to the ventilator failure caused by the internal and external environment during the use of the ventilator; electrical factors refer to breathing and failure caused by the change of power supply of key parts of the ventilator during the use of the ventilator. Air path coefficient refers to the ventilator itself to provide the user with oxygen and air negative feedback gas monitoring mode. While maintaining the stable gas supply function of the ventilator, the gas problem has a certain probability of causing the ventilator failure.

Figure 4 shows the experimental model of the ventilator. It can be seen that the humidity of the power module, the temperature of the air module, the pressure of the air source, the temperature of the air source, and the total load of the battery are all factors obtained from the rough reduction set. These factors are used as the input values for the input layer. The failure factors selected by the model (abnormal tidal volume, large deviation of oxygen concentration, failure of airtightness, and so on) were compared with the conventional failure factors.

(16) $$\begin{array}{c} \left\{\begin{array}{c} \text{Se}=\frac{1}{\max}\sum_{i=1}^{\max}\frac{{\text{TP}}_{i}}{{\text{TP}}_{i}+{\text{FN}}_{i}}\times 100\%,\\ \text{Sp}=\frac{1}{\max}\sum_{i=1}^{\max}\frac{{\text{TN}}_{i}}{{\text{TN}}_{i}+{\text{FP}}_{i}}\times 100\%,\\ \text{Acc}=\frac{1}{\max}\sum_{i=1}^{\max}\frac{{\text{TP}}_{i}+{\text{TN}}_{i}}{{\text{TP}}_{i}+{\text{FN}}_{i}+{\text{TN}}_{i}+{\text{FP}}_{i}}\times 100\%, \end{array}\right) \end{array}$$

where Se, Sp,  and Acc represent sensitivity, specificity, and accuracy, respectively; max is the total number of failure mode classification (max=3 is in research); TP is the true ratio; FP is a false positive case; FN is a false negative case; and TN means true negative.

## 3. Analysis of the Effect of Medical Imaging Equipment Health Evaluation and Fault Diagnosis

### 3.1. Effect Analysis of Health Evaluation of Medical Imaging Equipment Based on Neural Network

We select 96 groups of sampling data and select 75% of them as the training set and 25% as the test set; the corresponding characteristics of the three axial vibration signals are used as the network input, and the health of medical imaging equipment is used as the prediction output of the network. In frequency domain *A*^*∗*^, as the input parameter is combined with the single-layer network model based on DNN network, as model 1, select range feature *M*, *S*, *A*^*∗*^. As the input parameter is combined with the single-layer network model based on DNN network, as model 2, select range feature *M*, *S*, *A*^*∗*^. As the input parameter is combined with the single-layer network model based on DNN network, as model 3, the model proposed in this paper is based on the characteristics of amplitude range *M*, *S*, *A*^*∗*^. As input parameters are combined with the hybrid network model based on PLSR-DNN, the predicted values of the four models for the health degree of medical imaging equipment are shown in Figure 5.

As shown in Figure 5, compared with the actual health of medical imaging equipment corresponding to different sampling points, the health value of medical imaging equipment predicted by the proposed model is basically consistent with the actual health value. The difference between the predicted value and the actual value of health degree of medical imaging equipment in model 1 is the largest. Model 2 predicted the health degree of medical equipment, which was less than the actual health degree of medical equipment. The predicted value of medical imaging equipment in model 3 is basically consistent with the actual predicted value of medical equipment, but the predicted value of health degree of some medical imaging equipment is higher than the actual health value of medical equipment. The above results show that the proposed method is characterized by amplitude range *M*, *S*, *A*^*∗*^. As an input parameter, combined with the hybrid network model based on PLSR-DNN, it can achieve good application effect of medical imaging equipment health degree prediction, and the predicted value of health degree is basically consistent with the actual value of medical imaging equipment health degree.

In order to further explore the prediction effect of the four models, the prediction errors of the four models are studied and analyzed. The prediction error *E* is the difference between the actual health degree and the predicted health degree. When *E* > 0, the predicted health degree of the model is judged to be premature prediction; when *E* < 0, it was judged that the health degree predicted by the model was too late. The prediction errors of the four models are shown in Figure 6.

As shown in Figure 6, the prediction error of the proposed method based on PLSR-DNN hybrid network model is basically on the straight line of prediction error = 0, that is, the prediction error of the proposed method based on PLSR-DNN hybrid network model is basically 0 regardless of the specific location of the sampling point. When the sampling point is 20, the prediction error of model 1 is 150, and when the sampling point is 24, the prediction error of model 1 is −80. The prediction error of model 2 fluctuates greatly, and the predicted value of health degree of medical imaging equipment obtained at very few sampling points is consistent with the predicted value of actual health degree of medical equipment. The prediction error of model 3 fluctuates slightly around the error of 0, and the overall prediction error of model 3 is better than that of model 1 and model 2, but the overall effect is not as good as the proposed health evaluation method of medical imaging equipment based on PLSR-DNN hybrid network model.

### 3.2. Application Effect Analysis of Fault Diagnosis Method for Medical Imaging Equipment Based on Neural Network

In this study, 90 ventilator failures were selected as the training set, and the neural network was trained through the training set. There were 41 abnormal tidal volume failures, 22 abnormal oxygen concentration failures, and 27 abnormal air tightness failures in the training set. At the same time, the neural network training iterations are set to 1000 times. After the completion of the neural network training, the specific situation of BP neural network to identify the fault mode of medical imaging equipment is compared.

It can be seen from Figure 7 that in the training set, the detection results of the ventilator equipment fault training set in the training set by the proposed medical imaging equipment fault detection technology based on rough set and BP neural network algorithm show that the detection sensitivity, specificity, and accuracy of abnormal tidal volume fault are 87.7%, 75.6%, and 92.7%, respectively. The sensitivity, specificity, and accuracy were 90.9%, 95.5%, and 86.4%, respectively. The sensitivity, specificity, and accuracy of the method are 85.2%, 85.6%, and 92.6%, respectively. To sum up, it can be seen that when the medical imaging equipment fault detection technology based on rough set and BP neural network algorithm proposed in the study detects the training set, the total sensitivity of the corresponding ventilator fault detection is 87.8%, the corresponding specificity is 85.6%, and the accuracy rate is 91.1%.

After training, 60 ventilators were tested by using the rough set BP hybrid neural network. The test set was composed of 27 ventilators with abnormal tidal volume, 12 ventilators with abnormal oxygen concentration, and 21 ventilators with abnormal air tightness. The application effect of the proposed hybrid neural network based on rough set and BP is compared after training.

As shown in Figure 8, after training, the proposed medical imaging equipment fault recognition technology based on rough set and BP hybrid neural network has a recognition sensitivity of 70.4%, corresponding specificity of 85.2% for the ventilator with abnormal tidal volume, and an accuracy of 77.8% for the ventilator with abnormal tidal volume. In the number of malfunctioning ventilators with abnormal oxygen concentration, the recognition sensitivity, specificity, and accuracy of the medical imaging equipment fault recognition technology based on rough set BP hybrid neural network are 66.7%, 75.0%, and 83.3%, respectively. When the air tightness of the ventilator is abnormal, the recognition sensitivity, specificity, and accuracy of the medical imaging equipment fault recognition technology based on rough set BP hybrid neural network are 85.7%, 85.7%, and 95.2%, respectively. From the overall analysis, after training, the overall recognition sensitivity, specificity, and accuracy of the medical imaging equipment fault recognition technology based on rough set and BP hybrid neural network are 75.0%, 83.3%, and 85.0%, respectively.

## 4. Conclusion

The necessary link of medical imaging equipment management in health detection and fault detection is presented. Aiming at the health management of medical equipment, a health degree prediction technology based on PLSR-DNN hybrid network model is proposed. At the same time, a fault diagnosis technology based on rough set and BP neural network is proposed, and the practical application effect of these two technologies is analyzed. The results show that the predicted health value of different sampling points of medical imaging equipment is basically consistent with the actual health value of the medical imaging equipment based on PLSR-DNN hybrid network model, that is, the prediction error base between the predicted health value and the actual health value obtained by the technology is 0. In the training set, the overall recognition sensitivity, specificity, and accuracy of the proposed fault diagnosis technology of medical imaging equipment proposed by the rough set and BP neural network were 87.8%, 85.6%, and 91.1%, respectively. In the test set, the overall recognition sensitivity, specificity, and accuracy of the proposed fault diagnosis technology of medical imaging equipment proposed by the rough set and BP neural network were 75.0%, 83.3%, and 85.0%, respectively. The results show that the proposed health prediction technology based on PLSR-DNN hybrid network model and the fault diagnosis technology of medical imaging equipment based on rough set and BP neural network have good application effect in the health examination and fault diagnosis of medical equipment. Although some achievements have been made in this study, only ventilator is selected for the application test of medical imaging equipment fault diagnosis technology. The test results are not comprehensive. Other medical imaging equipment should be included in the analysis scope in the follow-up research.

## Figures and Tables

**Figure 1:** Health prediction model of PLSR-DNN hybrid neural network.

**Figure 2:** DNN model.

**Figure 3:** DNN model.

**Figure 4:** Experimental model building.

**Figure 5:** Comparison of actual health degree with the predicted results of four models.

**Figure 6:** Comparison of health prediction errors of four models.

**Figure 7:** Comparison of recognition results of ventilator fault pattern based on rough set and BP neural network in training set.

**Figure 8:** Comparison of results of ventilator fault pattern recognition based on rough set and BP neural network in test set.

**Table 1:** Rough set information of ventilator.

Ventilator brand and model	Oxygen supply concentration (%)	Does it affect respiratory therapy?
Hamilton C1	100	No
Delphi Evita4	74	Yes
…	…	…
Bird Vela	83	No

**Table 2:** Ventilator failure data collection.

Project	Mainly for	Acquisition module
Environmental data collection	Power supply module, air oxygen mixing module, and temperature and humidity data acquisition inside the cabinet	YC1001 temperature and humidity acquisition module collects 32 channels of independent temperature and humidity
Collection of electrical factors	Total load voltage and load current of ventilator, input voltage and current of turbine/compressor, voltage/current of air oxygen mixing module, and input voltage/current of exhalation/inhalation valve	16-channel JY-DAM1600AC module
Gas path factor collection	The pressure, concentration, and humidity of the input gas of the ventilator, the gas pressure at the input end of the air oxygen mixture, and the internal flow monitoring	LORA, YC1001 modular

## Data Availability

The data used to support the findings of this study are available from the corresponding author upon request.
